The article "IGST Combined with Conventional Drug Therapy and TCM Therapy for Treatment of Bilateral Vestibular Hypofunction" was retracted in 2023. Reasons: suspected computer-generated content; unreliable results or conclusions; concerns about the data; concerns about the results or conclusions.

# IGST Combined with Conventional Drug Therapy and TCM Therapy for Treatment of Bilateral Vestibular Hypofunction

**DOI:** 10.1155/2022/5689454

**Published:** 2022-06-07

**Authors:** Mingming Zhao, Jing Han, Liang Li

**Affiliations:** Department of Otolaryngology-Head and Neck Surgery, No. 2 Affiliated Hospital of Harbin Medical University, Harbin, Heilongjiang, China

## Abstract

**Objective:**

To investigate the effects of intensive gaze stability training (IGST) combined with conventional drug therapy and traditional Chinese medicine (TCM) therapy on hearing recovery and quality of life (QOL) in patients with bilateral vestibular dysfunction.

**Materials and Methods:**

A total of 120 patients with bilateral vestibular dysfunction admitted to our hospital from January 2019 to January 2020 were recruited and assigned to group A (*n* = 60) and group B (*n* = 60) based on the order of admission. Group B received conventional medication and TCM therapy, and group A received IGST plus conventional medication and TCM therapy. The serum biochemical indexes, blood rheology indexes, symptoms disappearance time, hearing recovery time, pure-tone hearing threshold, vestibular symptom index (VSI), and QOL of the two groups were compared.

**Results:**

The serum biochemical indexes and blood rheology indexes in group A were lower than those in group B after treatment (*P* < 0.001). Patients in group A had a shorter time lapse before symptoms disappearance and hearing recovery than those in group B (*P* < 0.001). Group A had lower results of the pure-tone hearing threshold (*P* < 0.001) and of VSI (*P* < 0.05) than group B. Patients in group A had higher QOL scores than those in group B after treatment (*P* < 0.001).

**Conclusion:**

IGST plus conventional drug therapy effectively improves the serum biochemical indexes and blood rheological indexes of patients with bilateral vestibular hypofunction, accelerates their hearing recovery process, and alleviates their clinical symptoms, thereby improving their QOL, which shows good potential in clinical application.

## 1. Introduction

When the bilateral vestibular function of the human body is impaired, patients may exhibit symptoms such as dizziness or hearing loss. In clinical practice, the activity of the inner and outer hair cells is reduced by weakening their excitability, which is conducive to restoring normal hair cell function and enhancing the patient's tinnitus sensation [1–3]. The hearing tinnitus comprehensive diagnostic instrument is commonly used for the treatment of bilateral vestibular hypofunction. However, patients show low treatment cooperation toward the instrument and its overall efficacy is modest [4–7]. The gaze stability training improves the vestibular locus coeruleus and visual condition and optimizes the maladaptive behavior of patients using physical training [8–11]. The body requires bilateral vestibular receptor information, visual information, and proprioceptive information afferents to maintain posture and balance. Impaired or damaged vestibular receptor function may lead to hearing loss, tinnitus, and vertigo in the organism [1]. Current clinical treatment focuses on the activation of the auditory efferent nervous system by masking sound, inhibiting the excitability and spontaneous activity of internal and external hair cells, and suppressing the lesioned central auditory nerve pathway to reduce or inhibit the perception of tinnitus [2, 3], which can effectively reduce the auditory efferent nervous system and thus achieve therapeutic benefits [4]. However, some patients showed poor compliance with this treatment method [5], and variations in treatment effects are attributed to patient tolerance and compliance. In recent years, an intensive gaze stability training (IGST) has been widely used in the treatment of patients with vestibular hypofunction. In traditional Chinese medicine, vestibular dysfunction is included in the categories of “vertigo,” “headache,” and “headwind,” with the disease located in the head orifice and the pathogenesis including wind, fire, phlegm, stasis, and deficiency. The head is the confluence of all yang. Wind, fire, phlegm, and stasis disturb the head orifices, and the deficiency of qi and blood and kidney essence causes dizziness and headache due to loss of nourishment of the medulla oblongata. The treatment lies in tonifying qi and blood, resolving phlegm, and quenching wind. Accordingly, this study recruited 120 patients with bilateral vestibular hypofunction that were admitted to our hospital from January 2019 to January 2020 to investigate the effect of IGST combined with conventional medication and traditional Chinese medicine (TCM) therapy on hearing recovery and QOL in patients with bilateral vestibular hypofunction.

The article "IGST Combined with Conventional Drug Therapy and TCM Therapy for Treatment of Bilateral Vestibular Hypofunction" was retracted in 2023. Reasons: suspected computer-generated content; unreliable results or conclusions; concerns about the data; concerns about the results or conclusions.

## 2. Information and Methods

### 2.1. General Data

A total of 120 patients with bilateral vestibular hypofunction admitted to our hospital from January 2019 to January 2020 were recruited and divided equally into group A (*n* = 60) and group B (*n* = 60) according to the order of admission. The two groups showed comparable patient characteristics (*P* > 0.05), as shown in Table 1. This study was approved by the hospital ethics committee.

### 2.2. Inclusion Criteria

Inclusion criteria of the patients in this study were as follows: (1) patients or their families had full knowledge of the study process and signed a consent form; (2) patients were diagnosed with bilateral vestibular hypofunction by combining medical history, examination results, and clinical manifestations [12–15]; (3) the time between onset and consultation was ≤2 weeks; (4) diagnostic criteria: with reference to the APTA Evidence-Based Clinical Practice Guideline: vestibular rehabilitation for peripheral vestibular hypofunction (2016) [6, 7], a comprehensive diagnosis was performed by combining the medical history, clinical manifestations, and caloric reflex test results. Clinical features of bilateral hypovestibular function include unstable walking in dark environments or on uneven surfaces and blurred vision during exercise or fast walking. During etiologic analysis, the patient had a clear history of transient ischemic attacks without hemiparesis, limb movement disorders, pathologic reflex signs, or other etiologies, and no lesions in the pontocerebellar horn or internal auditory tract were found on imaging.

### 2.3. Exclusion Criteria

Exclusion criteria for this study were as follows: (1) patients with psychiatric problems were incapable of communication; (2) patients with other organic diseases; (3) patients were diagnosed as inner auditory tract lesions or middle ear occupational lesions by imaging; and (4) patients with tinnitus symptoms before the onset of sudden deafness.

### 2.4. Methods

Group B received conventional medication and TCM therapy, and group A received IGST plus conventional medication and TCM therapy.

Conventional drug treatment: (1) patients received prednisone (Tianjin Lixiang Pharmaceutical Co., Ltd., State Pharmacopoeia H12020123) for 3 days at a dose of 1 mg/kg. (2) The patients with positive curative effects with prednisone were given medicine for 2 more days at the same dose; those with poor effects were discontinued and switched to intravenous 10 BU bacitracin injection (Beijing Tobishi Pharmaceutical Co., Ltd., State Pharmacopoeia H20030295) dissolved in 100 ml of 0.9% sodium chloride injection, twice daily. The duration of treatment was 5 days.

IGST: (1) gaze stability training: the patient was asked to keep both eyes open, shield one eye, and gaze horizontally forward with the other eye for 1 min. Two eyes were trained alternately for a total of 10 minutes. Eye movement was forbidden during the training. The training time was prolonged to 15 minutes after one day of training. (2) Visual tracking training: the patient needed to point out the positions on Schulte's square from the smallest one to the largest one and read out the number. The training lasted for 20 minutes. (3) Proprioceptive dependence training: the patient was asked to repeat the movements such as walking backward along the curve with eyes closed and skateboarding for 30 min.

The article "IGST Combined with Conventional Drug Therapy and TCM Therapy for Treatment of Bilateral Vestibular Hypofunction" was retracted in 2023. Reasons: suspected computer-generated content; unreliable results or conclusions; concerns about the data; concerns about the results or conclusions.

TCM dialectical therapy: the formula includes 10 g of Gastrodiae Rhizoma, 10 g of Uncariae Ramulus cum Uncis, 30 g of Haliotidis Concha (first decoction), 6 g of Chuanxiong Rhizoma, 10 g of Saposhnikoviae Radix, 10 g of Pinelliae Rhizoma, 15 g of poria, 15 g of Atractylodis Macrocephalae Rhizoma, 10 g of Viticis Fructus, 6 g of roasted liquorice root. Corydalis Rhizoma and Ligustici Rhizoma et Radix were added for severe headache, Caulis Polygoni Multiflori and Silktree Albizia Bark were added for insomnia, Polygoni Multiflori Radix and Rehmanniae Radix were added for liver and kidney deficiency, and Safflower and Peach kernel were added for blood stasis and obstruction. The above herbs were decocted twice in water to obtain 400 ml of filtrate, which was administered in the morning and evening before meals. The duration was treatment was 4 weeks.

### 2.5. Observational Criteria

1. Serum biochemical indexes include endothelin (ET), nitric oxide (NO), and superoxide dismutase (SOD). The comparison was conducted 30 days both before and after treatment.
2. Blood rheology indexes: whole blood viscosity (NS), whole blood viscosity at a high shear rate (NBH), and whole blood viscosity at a low shear rate (NBL) determined. The comparison was conducted 30 days both before and after treatment.
3. Time lapse before symptoms disappearance: symptoms included were tinnitus and vertigo, and the symptoms disappearance time of both groups of patients was compared.
4. Time lapse before hearing recovery: the time lapse before patients' hearing recovery was compared.
5. Pure-tone hearing threshold: the lightest sound that patients could precisely hear in both ears for different frequencies of pure-tones was detected. The lower the value, the better the patients' hearing. The time points of comparison were 30 days before and after treatment.
6. VSI: symptoms included balance, vertigo, dizziness, nausea, visual sensitivity, and headache, with a score between 0 and 10 points. The lower the score, the less severe the patient's symptoms. The time point of comparison was 30 days after treatment [16–19].
7. Quality of life (QOL): the QOL-C30 scale was used as the basis for scoring, which includes emotional function, physical function, social function, cognitive function, and role function. Higher scores were considered better QOL. The time point for comparison was 30 days after treatment [20–23].

### 2.6. Statistical Processing

SPSS 20.0 software was used for data analyses, and GraphPad Prism 7 (GraphPad Software, San Diego, USA) was used for graph plotting. Count data are analyzed using the chi-square test, and the measurement data were analyzed using the *t*-test. *P* < 0.05 means that the difference is statistically significant.

The article "IGST Combined with Conventional Drug Therapy and TCM Therapy for Treatment of Bilateral Vestibular Hypofunction" was retracted in 2023. Reasons: suspected computer-generated content; unreliable results or conclusions; concerns about the data; concerns about the results or conclusions.

## 3. Result

### 3.1. Serum Biochemical Indexes

The serum biochemical indexes in group A were lower than those in group B after treatment (*P* < 0.001), as shown in Table 2.

### 3.2. Blood Rheological Indexes

Group A had significantly lower blood rheological indexes after treatment than group B (*P* < 0.001), as shown in Table 3.

### 3.3. Symptom Disappearance

Patients in group A had a shorter time lapse before symptom disappearance than those in group B (*P* < 0.001) (Figure 1).

### 3.4. Hearing Recovery

Patients in group A had a shorter time lapse before hearing recovery as compared to group B (*P* < 0.001), as shown in Figure 2.

### 3.5. Pure-Tone Hearing Threshold Values

Group A had a better outcome of pure-tone hearing threshold values after treatment than group B (*P* < 0.001), as shown in Figure 3.

### 3.6. VSI

After treatment, VSI scores in group A were lower than those in group B (*P* < 0.05), as shown in Figure 4.

### 3.7. QOL

Patients in group A had higher QOL than those in group B (*P* < 0.001) (Table 4).

## 4. Discussion

Tinnitus is a common clinical symptom that is usually treated with medication to improve the patient's hearing by weakening the activity of the patient's hair cells and blocking the affected nerve pathways. However, the treatment compliance is considered poor due to its slow effect and higher recurrence [24–27]. In the present study, IGST was given to patients of group A based on drug treatment and results showed lower serum biochemical indexes and blood rheological indexes in group A than in group B after treatment (*P* < 0.001). Endothelin (ET) is an important indicator of the hypoxic state of a patient's inner ear cells. It facilitates vasoconstriction and when the elevation of its level is highly susceptible to cell necrosis. However, NO removes the newly emerged necrotic cells and an increase in NO leads to a rapid release of SOD that weakens oxygen-free radicals. IGST successfully stimulates the patients' brain cells, resulting in a sharp reduction in the frequency of excitotoxin secretion, the optimization of blood circulation after training [28, 29], and better serum biochemical indexes. The remarkably enhanced positive blood circulation and red blood cell deformation ability in patients of group A ensured a faster recovery from inner ear hypoxia and ischemia, as evidenced by the shorter time lapse before symptoms disappearance and better hearing recovery in group A than in group B (*P* < 0.001). In addition, IGST stimulates the inner ear nerve cells of patients to achieve a successful recovery with more satisfaction. As a result, group A with IGST intervention showed a lower pure-tone hearing threshold (*P* < 0.001) and a lower VSI (*P* < 0.05) after treatment as compared to group B. Consequently, patients in group A recovered faster with a superior treatment effect and had a higher QOL after treatment than group B (*P* < 0.001). The above results are consistent with the findings by Choi J S who proposed in his study that additional gaze stability training for patients in the experimental group based on medication treatment resulted in higher scores of physical function (73.21 ± 5.20), social function (59.16 ± 5.36), and role function (73.12 ± 6.21) than those in the control group (*P* < 0.001). This indicates that patients under the combination of treatment had a better QOL after treatment.

The article "IGST Combined with Conventional Drug Therapy and TCM Therapy for Treatment of Bilateral Vestibular Hypofunction" was retracted in 2023. Reasons: suspected computer-generated content; unreliable results or conclusions; concerns about the data; concerns about the results or conclusions.

The results of this study showed that there was a significant decrease in ET, NO, and SOD levels in both groups after treatment, and group A had significantly lower results, indicating the effectiveness of the treatment. Patients with vestibular hypofunction have an inadequate capillary blood supply to the inner ear [10, 11], and ischemia and hypoxia in cells cause a significant increase in the ET content. ET is a vasoactive substance that constricts blood vessels to aggravate hypoxia and cause cell necrosis, and NO is a main active substance of endothelium-derived diastolic factor that mediates cellular immunity and removes necrotic cells [12, 13]. Group A adopts IGST to improve and restore the vestibular function of the patient through daily training, which reduces the secretion of “excitatory” hormones and promotes vasodilatation and blood circulation. Therefore, the levels of ET, NO, and SOD decreased after treatment, which alleviates the local ischemia and hypoxia in the inner ear capillaries [14, 15].

In the present study, TCM therapy was used. According to TCM theory, vestibular dysfunction is attributed to the damage to the spleen and stomach qi, loss of spleen health, failure to transform water and grain essence and gathering of dampness and phlegm, and the blockage of phlegm and dampness, resulting in yin deficiency and internal wind, which disturbs the clear orifices and causes dizziness and headache [10]. In the TCM decoction used in the present study, Gastrodiae Rhizoma is the monarch medicine, which calms the liver and restores wind, settles fright, and calms the mind. Uncariae Ramulus cum Uncis and Haliotidis Concha are the ministerial medicines. Uncariae Ramulus cum Uncis clears heat, calms the liver, and settles panic, and Haliotidis Concha pacifies the liver, subdues yang, clears heat, and brightens the eyes. Chuanxiong Rhizoma invigorates blood and moves qi. Saposhnikoviae Radix disperses upper wind evil, overcomes dampness, and relieves pain. Pinelliae Rhizoma dries dampness, resolves phlegm, harmonizes the stomach, and stops vomiting. Poria nourishes the heart and tranquilizes the mind, strengthens the spleen, and permeates dampness. Atractylodis Macrocephalae Rhizoma strengthens the spleen, benefits the qi, dries dampness, and promotes water retention. Viticis Fructus disperses wind-heat and clears the head and eyes. Roasted liquorice root tonifies the earth and harmonizes the middle Jiao. Corydalis Rhizoma and Ligustici Rhizoma et Radix were added for headache to relieve pain, Caulis Polygoni Multiflori and Silktree Albizia Bark were added for insomnia, Polygoni Multiflori Radix and Rehmanniae Radix were added for liver and kidney deficiency, and Safflower and Peach kernel were added to invigorate blood circulation and remove blood stasis. The combination of all these herbs was effective in tonifying qi and blood, resolving phlegm, and quenching wind.

The article "IGST Combined with Conventional Drug Therapy and TCM Therapy for Treatment of Bilateral Vestibular Hypofunction" was retracted in 2023. Reasons: suspected computer-generated content; unreliable results or conclusions; concerns about the data; concerns about the results or conclusions.

## 5. Conclusion

In conclusion, IGST plus conventional drug therapy effectively improves the serum biochemical indexes and blood rheological indexes of patients with bilateral vestibular hypofunction and accelerates the disappearance of their symptoms and hearing recovery, which further ensures a better QOL for patients.

## Figures and Tables

**Figure 1:** Comparison of patients' symptom disappearance time (*x* ± *s*, d). *Note.* The horizontal axis of Figure 1 shows tinnitus and vertigo from left to right, respectively, and the vertical axis shows the time for the disappearance of symptoms (d); the black area in the figure is group A and the gray area is group B The disappearance time of tinnitus in group A was (8.42 ± 2.10) d and in the group B was (12.56 ± 2.14) d. The time taken for vertigo disappearance was (4.00 ± 1.24) d for group A and (6.54 ± 1.26) d for group B. ^*∗*^*P* < 0.05.

**Figure 2:** Comparison of patients' hearing recovery time (*x* ± *s*, d). The hearing recovery time was (7.23 ± 1.74) d for group A and was (10.59 ± 2.15) d for group B. ^*∗*^*P* < 0.05.

**Figure 3:** Comparison of pure-tone hearing threshold values of patients (*x* ± *s*, Hz). *Note.* The horizontal axis of Figure 3 from left to right is pretreatment and posttreatment, respectively, and the vertical axis is the pure-tone hearing threshold (Hz); the dotted line in the figure indicates group A and the straight line indicates group B. The pure-tone hearing threshold value before treatment was (88.26 ± 5.89) Hz in group A and (88.15 ± 5.45) Hz in group B. The pure-tone hearing threshold value after treatment was (68.52 ± 5.41) Hz in group A and (86.51 ± 5.14) Hz in group B. ^*∗*^*P* < 0.05.

The article "IGST Combined with Conventional Drug Therapy and TCM Therapy for Treatment of Bilateral Vestibular Hypofunction" was retracted in 2023. Reasons: suspected computer-generated content; unreliable results or conclusions; concerns about the data; concerns about the results or conclusions.

**Figure 4:** Comparison of VSI of patients after treatment (*x* ± *s*, points). *Note.*Figure 4 shows balance, vertigo, dizziness, nausea, visual sensitivity, and headache from left to right on the horizontal axis and VSI (score) on the vertical axis; the dotted line indicates group A and the squared line indicates group B. Posttreatment balance scores were (2.89 ± 1.21) in group A and (4.55 ± 1.22) in group B. Posttreatment dizziness scores were (2.78 ± 1.25) in group A and (3.56 ± 1.54) in group B. Dizziness scores after treatment were (2.10 ± 1.00) in group A and (4.02 ± 1.26) in group B. Posttreatment nausea scores were (1.05 ± 0.51) in group A and (1.89 ± 0.54) in group B. Visual sensitivity scores after treatment in group A were (1.44 ± 1.01) and in group B (2.99 ± 1.24). Posttreatment headache scores were (1.55 ± 1.22) in group A and (1.98 ± 1.01) in group B. ^*∗*^*P* < 0.05.

**Table 1:** Comparison between the general data of the patients.

Groups	Group A (*n* = 60)	Group B (*n* = 60)	*X* ^2^/*t*	*P*
Gender			0.035	0.853
Male	25	24		
Female	35	36		
Mean age (years)	55.21 ± 6.20	55.23 ± 6.21	0.018	0.986
Types of disease				
Low-frequency descending	15	14	0.046	0.831
High-frequency descending	31	32	0.033	0.855
Flat-frequency descending	14	14	—	>0.05
BMI (kg/m^2^)	22.01 ± 1.52	21.89 ± 1.53	0.431	0.667
MARS-A scores	14.88 ± 2.54	14.89 ± 2.56	0.021	0.983

**Table 2:** Comparison of serum biochemical indexes of patients (*x* ± *s*).

Groups	ET (pg/ml)		NO (*μ*mol/L)		SOD (nU/ml)	
	Before treatment	After treatment	Before treatment	After treatment	Before treatment	After treatment
Group A	72.15 ± 5.89	51.56 ± 5.56	56.78 ± 5.25	30.56 ± 4.51	82.11 ± 4.58	52.12 ± 5.47
Group B	72.52 ± 5.45	62.78 ± 5.68	56.88 ± 5.23	41.56 ± 4.57	82.56 ± 4.12	69.15 ± 4.88
*T*	0.357	10.934	0.105	13.271	0.566	17.995
*P*	0.722	<0.001	0.917	<0.001	0.573	<0.001

**Table 3:** Comparison of patients' blood rheological indexes (*x* ± *s*, mPa-s).

Groups	NS		NBH		NBL	
	Before treatment	After treatment	Before treatment	After treatment	Before treatment	After treatment
Group A	2.20 ± 0.45	1.11 ± 0.21	6.45 ± 1.21	3.32 ± 1.10	10.36 ± 2.78	7.11 ± 2.14
Group B	2.21 ± 0.39	2.01 ± 0.23	6.42 ± 1.35	5.10 ± 1.45	10.39 ± 2.59	8.99 ± 2.54
*T*	0.130	22.384	0.128	7.576	0.061	4.385
*P*	0.897	<0.001	0.898	<0.001	0.951	<0.001

**Table 4:** Comparison of QOL of patients after treatment (*x* ± *s*, points).

Groups	Emotional function	Physical function	Social function	Role function	Cognitive function
Group A	66.21 ± 5.58	72.56 ± 5.23	59.56 ± 5.14	72.12 ± 6.23	85.11 ± 5.89
Group B	60.11 ± 5.45	62.89 ± 5.21	52.12 ± 5.23	59.89 ± 6.54	78.54 ± 5.88
*t*	6.058	10.146	7.859	10.488	6.115
*P*	<0.001	<0.001	<0.001	<0.001	<0.001

The article "IGST Combined with Conventional Drug Therapy and TCM Therapy for Treatment of Bilateral Vestibular Hypofunction" was retracted in 2023. Reasons: suspected computer-generated content; unreliable results or conclusions; concerns about the data; concerns about the results or conclusions.

## Data Availability

All data generated or analyzed during this study are included in this published article.
